The article "Value of 3D Printed PLGA Scaffolds for Cartilage Defects in Terms of Repair" was retracted in 2023. Reasons: signs of a paper mill; suspected computer-generated content; unreliable results or conclusions; concerns about the data.

# Value of 3D Printed PLGA Scaffolds for Cartilage Defects in Terms of Repair

**DOI:** 10.1155/2022/3561430

**Published:** 2022-08-03

**Authors:** Longkun Fan, Wei Teng, Jinqiu He, Dongni Wang, Chunhui Liu, Yujia Zhao, Limin Zhang

**Affiliations:** ^1^Cangzhou Central Hospital, No. 16, Xinhua West Road, Cangzhou City, Hebei Province, China; ^2^Cangzhou Women and Children's Health Hospital, Fuyang North Avenue, Cangzhou City, Hebei Province, China

## Abstract

**Objective:**

To examine the poly (lactic-co-glycolic acid) and sodium alginate (SA) scaffolds produced by 3D printing technology, access the healing morphology of bones following PLGA/SA implantation within rat cartilage, and examine osteogenesis-related factors in rat serum to determine the efficacy of PLGA/SA scaffolds in healing animal cartilage injuries. To identify the potential of this material to repair a tissue engineering osteochondral injury.

**Methods:**

Polylactic acid-glycolic acid copolymer and sodium alginate were used as raw materials to create PLGA/SA scaffolds. We observed the scaffold's macrostructure and microstructure, and the scaffold's microstructure was observed through a scanning electron microscope (SEM). The mechanical toughness of a stent was assessed using a biomechanical device. Hematoxylin-eosin staining revealed immune rejection after embedding the scaffolds under the skin of SD rats. The CCK-8 cell proliferation test kit was used to measure cell proliferation. An experimental model of cartilage injury in the knee joint was created in rats. Rats were used to establish an experimental model of cartilage damage in the knee joint. 120 female rats aged 5 weeks were chosen at random from the pool and divided into the experimental and control groups. They were all completely anesthetized with an anesthetic before having the lateral skin of the knee articular cartilage incised. Implanted PLGA/SA scaffolds were not used in the control group and only in the experiment group. Both groups of rats had their muscles and skin sutured and covered in plaster bandages. On the third, seventh, fourteenth, twenty-first, twenty-eighth, and thirty-fifth days after the procedure, the two groups of rats were divided into groups. At various stages, bone tissue, blood samples, and cartilage were examined and evaluated. Immunohistochemistry was used to identify the local bone morphogenetic protein-2 (BMP2).

**Results:**

(1) PLGA/SA was successfully used to build an artificial cartilage scaffold. (2) Macroscopic and SEM observation results showed the material had increased density and numerous microvoids on the surface. (3) The result of the biomechanical test showed that the PLGA/SA scaffold had superior biomechanical characteristics. (4) The stent did not exhibit any noticeable immunological rejection, according to the results of the subcutaneous embedding experiment performed on rats. (5) The CCK-8 data demonstrated that as the cell development time rose, the number of cells gradually increased. However, there was not statistically significant difference between the growth of the cells in the scaffold extract and the control group (*P* > 0.05). (6) A successful rat model based on a cartilage defect of the medial knee joint has been built. (7) Observations of specimens revealed that the experimental group's bone tissue score was higher than that of the control group. (8) Using immunohistochemistry, it was found that the experimental group's BMP2 expression was higher on the 7th, 14th, and 28th days than it was in the control group (*P* < 0.05).

The article "Value of 3D Printed PLGA Scaffolds for Cartilage Defects in Terms of Repair" was retracted in 2023. Reasons: signs of a paper mill; suspected computer-generated content; unreliable results or conclusions; concerns about the data.

**Conclusion:**

Strong mechanical and biological properties are present in stable, biodegradable PLGA/SA scaffolds that mimic cartilage. We demonstrated that the cartilage biomimetic PLGA/SA scaffold may repair cartilage and prevent negative reactions such as osteoarthritis in rat knee cartilage, making it suitable as a cartilage scaffolding material for tissue engineering. The PLGA/SA scaffold was also able to promote BMP2 expression in the bone healing zone when inserted into a knee cartilage lesion. Improved cartilage damage is the outcome of BMP2's promotion of bone formation and restriction of bone resorption in the bone healing zone.

## 1. Introduction

Common causes of articular cartilage (AC) injuries include sports-related injuries, accidents, and joint conditions [1]. The quality of life for the patient is decreased by the severe knee pain, edema, and joint stiffness caused by AC injuries. Furthermore, cartilage's capacity for self-repair is significantly diminished since it lacks lymphatic circulation, nerve tissue, and a blood supply when wounded [2, 3]. Osteoarthritis will occur from prolonged cartilage damage because it will influence the subchondral bone [4]. This makes it very challenging to cure cartilage damage [5]. Currently, a variety of therapies are used in clinical settings, such as chondrocyte transplantation, autologous and allogeneic cartilage transplantation, and periosteal stimulation. However, these therapies are expensive and have a poor success rate, making them unsuitable for patient needs [6, 7]. As a result, we are constantly searching for a better options. Alginate offers the stability, solubility, viscosity, and safety parameters needed to be utilized as an excipient in medicinal compositions, according to scientific investigations. It has been utilized in tissue engineering as a natural polysaccharide produced from brown algae, such as kelp, as a cartilage substitute [8, 9]. Studies have demonstrated that sodium alginate makes a great natural scaffold. Because of its intrinsic biocompatibility and gel-like characteristics, sodium alginate can maintain chondrocyte form. A sodium alginate scaffold can be used to cure cartilage damage, as demonstrated by Schoolten et al. in their research [10]. Acid saline gel has been utilized successfully to regenerate cartilage from dental pulp stem cells (HDPSCs) and has been shown to be efficient [11]. Interestingly, Mata et al. discovered that sheep and rabbits could promote chondrogenesis using biphasic sodium alginate scaffolds [12]. We use both natural and biodegradable components because using simply natural materials cannot guarantee the scaffold's internal stability. The four most popular 3D printing technologies currently used in clinical settings are low-temperature deposition manufacturing (LDM), light-curing stereolithography (SLA), fused deposition modeling (FDM), and selective laser sintering (SLS) [13]. LDM 3D printing technology was selected for this study.

The article "Value of 3D Printed PLGA Scaffolds for Cartilage Defects in Terms of Repair" was retracted in 2023. Reasons: signs of a paper mill; suspected computer-generated content; unreliable results or conclusions; concerns about the data.

The composition ratio of PGA and PLA can be used to calculate the degradation rate of PLGA, which is created when polyglycolic acid and PLA are polymerized. Because of their outstanding biocompatibility, degradability, and superior mechanical qualities, PLGAs are frequently utilized in scaffold construction and have received FDA approval for clinical applications. However, because PLGA is hydrophobic and lacks sites for cell identification and attachment, this interferes with the material's affinity, and as a result, the adhesion and development of cells on the surface. This problem has led to attempts to include PLGA into various organic and inorganic materials to enhance the performance of composite scaffolds [14, 15]. The mechanical strength and strain tolerance of a bioactive scaffold created using LDM 3D printing ensure that the microscopic structure of the organism will not be harmed in the interest of reproducibility [16]. Therefore, we anticipate that the capabilities of PLGA and SA will be complemented by their combination, with PLGA acting as the scaffold's main component to give strong mechanical strength and biocompatibility. The two together offer more hydrophilic sites for cell attachment and improve the composite scaffold's mechanical strength, while silicon encourages the production of cartilage matrix to create a scaffold material that is better suited for the use of cartilage tissue engineering using LDM [17]. The purpose of this study is to determine whether cartilage damage in rats may be effectively treated with PLGA/SA.

The article "Value of 3D Printed PLGA Scaffolds for Cartilage Defects in Terms of Repair" was retracted in 2023. Reasons: signs of a paper mill; suspected computer-generated content; unreliable results or conclusions; concerns about the data.

## 2. Materials and Methods

### 2.1. Main Materials and Reagents

The main materials and reagents are given in Table 1.

### 2.2. Laboratory Animals

Complete medium for lab rats (Shandong Qingdao Laboratory Animal Co. Ltd.) was made up of the following ingredients: DMEM High Glucose Basal Medium (Gibco, USA), 10% fetal bovine serum (Gibco, USA), and 1% double antibody (Gibco, USA). The Cangzhou Central Hospital Ethics Committee gave its approval to the study protocol prior to enrollment. Approval number: HS-DJS20200224.

### 2.3. Experimental Methods

#### 2.3.1. Preparation of Bioactive Scaffolds

A 3D bionic printer was used to fabricate PLGA/SA scaffolds. Until all of the particles were dissolved, we continuously mixed 10 g of PLGA powder and 2.5 g of SA powder for 18 hours at 25°C. The acquisition of PLGA/SA scaffold material was the last stage. A PLGA/SA 3D printed bone scaffold was produced using a 3D bionic printer A that was outfitted with an ink cartridge that allowed molten materials to be sprayed in the 3D direction in accordance with predefined specifications.

#### 2.3.2. Animal Surgery Procedure

120 healthy adult rats were used for the study, and they were randomly split into two groups: an experimental group and a control group (Table 1). To produce anesthesia, an intramuscular injection of 2 percent pentobarbital sodium (0.3 ml/100 g) was given to the experimental group. The skin and subcutaneous tissue were incised sequentially from the medial incision of both lower extremities' knee joints, exposing the joint capsule, entering the joint cavity, and fully exposing the trochlea of the femur. On both femurs, a drill was used to create a 4 mm long, full-thickness bone defect that reached the medullary cavity in the proximal third of the trochlea. When the cartilage defect model was finished, the sterilized PLGA/SA scaffold was pressed and implanted, whereas the blank group was simply sutured. We gave the experimental animals complete reign to go about after they were woken from anesthesia. Penicillin was administered to prevent infection, the femur was bandaged, and erythromycin ointment was applied to the incision for three days following surgery (see Table2).

#### 2.3.3. Specimen Collection

The rats were sacrificed by blood draw from the abdominal aorta on days 3, 7, 14, 21, 28, and 35 following intraperitoneal anesthesia. The femurs of 10 rats from each group—10 from the experimental group and 10 from the control group—were removed, and the bone density of each group's femurs was assessed. All of the rats' blood was collected, and samples were examined.

#### 2.3.4. Bone Tissue Score

O'Driscoll's histological scoring system was used to assess the results of cartilage repair. The evaluation takes into account the structural makeup of the cells, their morphology, and the degree of degeneration and fusion of the repaired tissue with the surrounding tissue.

The article "Value of 3D Printed PLGA Scaffolds for Cartilage Defects in Terms of Repair" was retracted in 2023. Reasons: signs of a paper mill; suspected computer-generated content; unreliable results or conclusions; concerns about the data.

#### 2.3.5. Immunohistochemical Detection of BMP2

We immersed sections of dewaxed paraffin in water. The nuclei were dehydrated, mounted, and seen under a microscope after being counterstained with hematoxylin; images were then gathered and evaluated. The cumulative optical density (COD) and the tissue pixel area (AREA) for the image were calculated using at least five fields of view at 200× that were randomly chosen in each sector. The average optical density (AOD) value was then determined using the formula AOD = COD/AREA; the higher the AOD value, the stronger the positive expression.

### 2.4. Statistical Analysis

SPSS22.0 was used for the statistical analysis, which included the following data analysis: measurement data were expressed as mean ± standard deviation, and a *t*-test was conducted; count data were expressed as a percentage, and a chi-square test was performed. The cutoff for statistical significance was 0.05.

## 3. Results

### 3.1. An Overview of the Conditions for Sampling Experimental Animals

The experimental animals all grew healthily, despite an infection that claimed the lives of two rats, and all of the experimental animals grew well. No evident inflammatory secretions, synovial hyperplasia, or tissue adhesion between the synovium and surrounding tissues were present.

### 3.2. Specimen Collection and Observation

GraphPad Prism 5 was used to analyze the data and determine how well each experimental group's subchondral bone growth was measured by the bone volume fraction (Table 3). At 21 and 35 days, the experimental group's cartilage growth was substantially faster than that of the control group, and the PLGA/SA stent group's bone volume percentage was significantly larger than that of the control group (*P* < 0.05).

### 3.3. Histological Scoring

To evaluate and compare the repair effectiveness of cartilage defects between the two groups, a histological grading method was employed. 14 days following the procedure, the experimental group scored 8.6 ± 2.2, whereas the control group scored 7.6 ± 1.7. Statistical analysis revealed that the experimental group outperformed the control group by a statistically significant margin (*P* < 0.05). There was a statistically significant difference between the experimental and control groups at 28 and 35 days following surgery, with the experimental group scoring higher than the control group (*P* < 0.05) (Table 4).

The article "Value of 3D Printed PLGA Scaffolds for Cartilage Defects in Terms of Repair" was retracted in 2023. Reasons: signs of a paper mill; suspected computer-generated content; unreliable results or conclusions; concerns about the data.

### 3.4. Results of BMP2-Positive Rate

Figure 1 shows immunohistochemical staining images (positive rate analysis results of BMP2), which show that the local BMP2 levels had increased in both the experimental and blank groups and that the experimental group had been statistically and significantly superior to the control group on the 7th, 21st, and 35th days (*P* < 0.05).  Figure 2 shows how PLGA mediates the action of bone morphogenetic proteins.

## 4. Discussion

The ability of cartilage to repair itself once it has been injured is quite limited due to the lack of blood supply to the cartilage itself, which makes cartilage defects a prevalent clinical problem. Since the concept of tissue engineering was created, more and more study has been focused on using these approaches to address the issue of cartilage defects [18]. Bone development is one of the more significant therapeutic applications of 3D printing technology [19]. In addition to providing quick turnaround times, high repeatability, accuracy, level of control, and the capacity to create personalized scaffolds, 3D printing also has the ability to alter the composition of scaffolds to enhance their performance [20]. The ideal scaffold material is one of the most important elements in tissue engineering to enable tissue regeneration. The following characteristics should be present in scaffolds that can support tissue engineering applications: (1) it has excellent hydrophilic properties and biocompatibility; (2) it has a regular three-dimensional high porosity structure with interconnected pores, which facilitates cell migration on the scaffold, extracellular nutrient exchange and transport of cellular waste, etc.; (3) the material is degradable and the rate is easily controlled; (4) its mechanical properties are sufficient to support the skeleton. Skeletal support for cell growth and tissue generation can be provided by the scaffold material's three-dimensional spatial structure and superior mechanical strength. The scaffold's hydrophilic properties and biocompatibility promote cell colonization and growth, while its high porosity promotes oxygen and nutrient delivery, cell movement, and angiogenesis [21, 22].

In our study, this method was used to create porous PLGA/SA scaffolds that integrated the benefits of both PLGA and SA [23, 24]. The bone tissue composition research revealed that the PLGA/SA scaffolds had excellent biocompatibility, biodegradability, and bone induction characteristics. Furthermore, it might increase cell adhesion to the scaffold surface as well as proliferation. Seven days after surgery, the scaffold started to break down, releasing nutrients for bone development. As early as day 14, the bone tissue strength of the experimental group was significantly higher than that of the control group. The difference was much more pronounced on day 28, showing that PLGA/SA promoted bone tissue to a relatively high level of strength; this is crucial for lowering the risk of early fractures. The synthetic polymer PLGA may be the main cause because it has good plasticity and biocompatibility, and because it can be combined with other materials to enhance the “discrete and reinforcing” effect of silicon particles and boost their own particle strength, thereby increasing the composite's mechanical strength [25]. More research suggests that the material has a positive osteogenic effect. The experiment's findings revealed considerable variations in BMP2's positive indications, which are a measure of quick bone remodeling. Since it is a potent inducer of osteoblast proliferation and differentiation [26], the bone morphogenetic protein 2 (BMP2) is crucial in promoting vascularization [27]. The technique has gradually been used for spinal fusion and the treatment of clinical bone tissue defects [28].

The article "Value of 3D Printed PLGA Scaffolds for Cartilage Defects in Terms of Repair" was retracted in 2023. Reasons: signs of a paper mill; suspected computer-generated content; unreliable results or conclusions; concerns about the data.

At this time, bone formation was more active in the experimental group than in the control group, showing that the PLGA-SA scaffold can activate BMP2 to promote bone factor (Figure 2) and improve cartilage injuries. This cytokine, like the majority of cytokines, has a very short half-life in the body, which is a typical drawback of cytokines. In order to achieve long-term improvements in nerve repair, it is therefore still challenging for contemporary researchers to connect tissue engineering scaffolds and release them over a protracted period of time [29]. We draw the conclusion that 3D-printed PLGA/SA scaffolds can successfully promote cartilage repair and have a significant impact on cartilage repair based on the findings discussed above.

There are still several issues to be resolved even though this experiment offers some reference values for the repair of cartilage defects by 3D-printed PLGA scaffolds: (1) future in vitro degradation experiments must investigate the two scaffolds' in vitro degradation rate and nature of the degradation products; (2) more animal studies are required to determine how the two scaffolds affect cartilage repair.

## 5. Conclusion

This research demonstrates that the improved performance of bioengineered PLGA/SA scaffolds as cartilage scaffolds, which can both increase cartilage osteogenic activity and decrease bone absorption. Calcium and phosphorus are released during the scaffold's degradation, and they later convert into raw materials. The PLGA/SA scaffold can also regulate BMP2, an essential protein involved in bone healing to promote osteogenesis. This highlights how important this scaffold is for treating cartilage damage and how it can help individuals with cartilage injury function better while also making following rehabilitative therapy less challenging.

The article "Value of 3D Printed PLGA Scaffolds for Cartilage Defects in Terms of Repair" was retracted in 2023. Reasons: signs of a paper mill; suspected computer-generated content; unreliable results or conclusions; concerns about the data.

## Figures and Tables

**Figure 1:** Immunohistochemical BMP2-positive rate results.

**Figure 2:** PLGA mediates bone morphogenetic proteins.

**Table 1:** Main materials and reagents.

Reagent name	Origin and company name
Polyglycolic acid	Beijing Chemical Reagent Co. Ltd., China
Polyglycolic acid	Beijing Chemical Reagent Co. Ltd., China
Polyglycolic acid	Nanjing Jiancheng Biological Company, China
Pentobarbital sodium injection	Beijing Chemical Reagent Co. Ltd., China
HE dye kit	Nanjing Jiancheng Biological Company, China
Anhydrous ethanol	Nanjing Jiancheng Biological Company, China
Penicillin injection powder	Nanjing Jiancheng Biological Company, China

**Table 2:** Grouping of experimental animals.

	Experimental group (PLGA/SA scaffold group)	Blank group (no stent implantation group)
3 days after surgery	10	10
7 days after surgery	10	10
14 days after surgery	10	10
21 days after surgery	10	10
2 to 8 days after surgery	10	10
3 to 5 days after surgery	10	10

**Table 3:** Evaluation of the growth of subchondral bone in each experimental group.

	Experimental group (PLGA/SA scaffold group)	Blank group (no stent implantation group)
3 days after surgery	0.329213	0.249217
7 days after surgery	0.369251	0.289311
14 days after surgery	0.390928	0.352201
21 days after surgery	0.429224	0.375234
2 to 8 days after surgery	0.599286	0.413352
3 to 5 days after surgery	0.619262	0.476624

**Table 4:** Histological score statistics.

Group/time	3 days	14 days	21 days	28 days	35 days
Blank group	7.3 ± 1.4	7.6 ± 1.7^*∗*^	8.2 ± 1.2	8.3 ± 1.5^*∗*^	8.5 ± 2.4^*∗*^
Experimental group	7.3 ± 2.1	8.6 ± 2.2^*∗*^	8.6 ± 2.4	9.1 ± 1.1^*∗*^	10.6 ± 2.1^*∗*^

^*∗*^Statistically significant difference.

## Data Availability

No data were used to support this study.
